The article "Analyzing the Relationship between Hotel Brand Image, Service Quality, Experience Marketing, and Customer Satisfaction under the Environment of Social Network" was retracted in 2023. Reasons: unreliable results or conclusions; concerns about the data; concerns about the peer review; concerns about the citations.

# Analyzing the Relationship between Hotel Brand Image, Service Quality, Experience Marketing, and Customer Satisfaction under the Environment of Social Network

**DOI:** 10.1155/2022/1064712

**Published:** 2022-07-30

**Authors:** Wen Xi

**Affiliations:** Department of Management, Taiyuan Normal University, Taiyuan 030600, China

## Abstract

Based on the development background of the social network environment, higher requirements are put forward for the development and transformation of hotels in the new era. As a representative industry in the service industry, the service quality and experience provided by the hotel can meet the feelings and needs of customers. According to the data of the hotel industry in previous years, it can be found that from 2015 to 2018, the average revenue of hotel rooms available for rent (RevPAR) decreased by 7.7%, 5.3%, and 7.7%, respectively; The occupancy rate dropped to the lowest point at the end of 2018 and then began to rise gradually. In addition, while the economy recovers, the tourism industry has driven the hotel industry. RevPAR has increased by—1.4% and 3.5% year-on-year, and the occupancy rate has increased by 3.6% and 2.0% year-on-year. In 2018, China's star hotels generally showed an upward trend. This also shows the attraction of hotel brand logo to customers. By studying the factors such as brand image and service quality, we can establish the viscosity with customers. This paper explores the relationship between various elements and customers and puts forward effective suggestions in order to further improve the service level of the hotel.

## 1. Introduction

Based on the social network environment, this paper explores the relationship between the hotel and customers from the supply side and starts from the aspects of customer satisfaction and emotion so as to provide new methods to improve the service quality of the hotel and provide a new path for the development of the hotel. Based on the dimensions of community experience, such as hotel brand and service quality, as well as the impact of user experience, this paper draws a comprehensive conclusion [1]. The research conclusion points out that we should focus on improving the brand, service, and quality of the hotel, strengthening the community interaction experience, consolidating the brand community information experience, promoting user immersion, establishing an important element of long-term contact between the hotel and customers, and ensuring customers' loyalty to the hotel brand.

The study of social networks originated in the 1930s. Structure is the relationship between various parts of the whole. Therefore, the concept of social structure naturally includes the relationship between various parts of human society. Therefore, social structure refers to the network of actual social relations, which is the sum of all individual social relations at a specific time. With the rapid development of the Internet, the communication between people has gradually shifted from reality to network, and the virtual community has become an integral part of people's life (as shown in Figure 1). The platform follows common norms and carries out online interaction around common interests, needs, or purposes. People can exchange product or service information, comment, or suggestions through virtual communities. Later, on the basis of the two, the virtual brand community gradually appeared [2, 3].

The article "Analyzing the Relationship between Hotel Brand Image, Service Quality, Experience Marketing, and Customer Satisfaction under the Environment of Social Network" was retracted in 2023. Reasons: unreliable results or conclusions; concerns about the data; concerns about the peer review; concerns about the citations.

According to the analysis, the value cocreation theory in the field of marketing has gradually attracted the attention of the academic circles because of its distinctive characteristics of the times and universal applicability and has been introduced into many research fields. More and more researchers have begun to pay attention to the problem of tourism experience value cocreation. On the basis of traditional understanding, these existing research results have promoted the theoretical and practical research of experience, both in terms of ideas and technology: first, rerecognize the role of tourists in tourism activities and their role in tourism experience value and point out that tourists are not only consumers of tourism services, but also participate in the process of creating tourism experience value through their own resource investment; Second, it carried out empirical research from the perspective of customers and enterprises, respectively, laying a foundation for theoretical exploration and practical research on customer experience creation under the new social situation and the background of the times [4].

## 2. Literature Review

In academia, experience has attracted the attention of scholars in different disciplines from a very early time, but the definition of experience has different emphases, so it is difficult to give a recognized and consistent definition. In the field of psychology, the definition of experience is developed on the basis of “flow experience” [5, 6]. “Flow experience” is the overall feeling of an individual's whole-hearted concentration on an activity, which is the process of optimal experience. It is a need that is continuously deepened through emotional and spiritual upward and belongs to the overall perception set of the individual.

In previous studies, due to the different research backgrounds of scholars, the meaning of customer experience is often different, and the measurement dimensions used are also different, but the dimensions used more frequently include: sensory, emotion, thinking, action, related experience, and so on. However, so far, the measurement dimension of customer experience is still controversial. Based on the one-dimensional perspective, some scholars believe that starting from the customer network experience, they propose that the customer experience is composed of usability experience. The two-dimensional perspective is based on the industrial background, emphasizing a variety of sensory behaviors pursued by customers' experience, stimulating customers' emotion and cognition so as to obtain more consumption intention. The three-dimensional perspective is to analyze the comprehensive feelings of customer experience, which is composed of perception, emotion, and social experience. It is a comprehensive response and cognition caused by the interaction with the consumption process and hotel. As a perspective, it studies the interaction of customer experience, service value, and other experiences. Customer experience is a process in which consumers' needs are continuously met in the consumption situation provided by enterprises. It is a four-dimensional structure composed of products, services, emotions, and social experiences. Customer experience is a kind of tourists' feeling and comprehensive evaluation of the humanities, society, image, and other aspects of the tourism destination. The five-dimensional perspective is to further brand customer experience. Customer experience is a series of feelings such as cognition and impression generated by tourists in the service consumption scenario provided by enterprises, including function, sensory, emotional, social, and knowledge experience. Hsu and Tsou believe that customer experience refers to the feeling generated by blog users when browsing content and is composed of five dimensions: sensory, sensory, thinking, behavior, and related experience [7–9].

The article "Analyzing the Relationship between Hotel Brand Image, Service Quality, Experience Marketing, and Customer Satisfaction under the Environment of Social Network" was retracted in 2023. Reasons: unreliable results or conclusions; concerns about the data; concerns about the peer review; concerns about the citations.

Some scholars have studied the impact of social impact theory on consumer behavior. In the social circle of friends, through the role of identification and internalization mechanism, consumers' purchase intention can be affected. When consumers are in a certain community or circle, other people in the community or circle have an impact on their attitudes and behaviors. Some scholars believe that innovation diffusion mainly includes five processes: awareness, persuasion, decision, implementation, and confirmation. Some factors will affect the acceptance level of personal new things. Such as comparative advantage and observability. Comparative advantage describes the degree to which an individual's advantage in using innovation is better than that of not using it. Compatibility refers to the matching degree between an individual's own values, ideas, etc., and the connotation of innovation. The higher the matching degree, the more likely an individual is to accept innovation. Complexity is the difficulty of individual understanding and adopting innovation. The lower the complexity, the faster the acceptance. Testability describes the level of innovation that can be tested. High testability can reduce the uncertainty of individual perception, and the faster innovation is accepted. Observability is that if the innovation results can be seen by others and can be spread among friends and people in some ways, they will be more easily accepted [10].

## 3. Model Construction

To explore the impact of different dimensions of experience value on satisfaction based on online comments, we first need to elaborate the definition of experience value and the connotation of customer satisfaction in combination with previous research results, then introduce emotion analysis technology, and then analyze the relationship between experience value and customer satisfaction based on online comment data in combination with cognitive evaluation theory and stimulating organism response theory.

### 3.1. Experience Value

First of all, as far as its main body is concerned, experience value is the expression of customers' subjective feelings in the process of consumption; Secondly, as far as its production process is concerned, experience value is a comprehensive perceptual evaluation that runs through the whole process of customer consumption experience and is not limited to a certain stage or a certain perceptual level; Finally, in terms of its trigger mechanism, experience value is formed in the direct or indirect interaction process between consumers and products and services. It is a complex and changeable feeling or perception state, which can effectively improve the satisfaction level of consumers and establish the competitive advantage of enterprises, as shown in Figure 2.

As shown in Figure 3, in the model, customer experience is the prevariable of brand loyalty. Brand loyalty is divided into two dimensions: behavior and attitude loyalty, and customer consumption (CS) is introduced to expand this framework [11, 12]. Measured by consumers' share of purchases of a particular brand relative to overall usage or spending on products in the same category. Results show that customer experience positively affects attitudinal and behavioral loyalty.

In order to explore the formation mechanism of brand loyalty, Bilgihan conducted a questionnaire survey on 2500 website consumers and established and tested a comprehensive model of influencing factors of customer loyalty of hotel reservation websites (as shown in Figure 4 below). The results show that trust has the greatest impact on consumers' online shopping intention, and the hedonic and utilitarian characteristics of the website will positively affect consumers' immersion and then affect their loyalty.

The article "Analyzing the Relationship between Hotel Brand Image, Service Quality, Experience Marketing, and Customer Satisfaction under the Environment of Social Network" was retracted in 2023. Reasons: unreliable results or conclusions; concerns about the data; concerns about the peer review; concerns about the citations.

### 3.2. Customer Satisfaction

Customer satisfaction is regarded as the evaluation of consumers' cumulative feelings after purchase behavior, which is the overall evaluation of purchase and consumption experience for a period of time after purchase [13]. The model of customer satisfaction is shown in Figure 5, and different psychological changes will occur according to the actual consumption feeling.

Applying cognitive evaluation theory to the research of this paper produces the following thoughts: first, in the composition of hotel experience value of customers, including the external motivation of hotel tenants, that is, corresponding to the practical value mentioned in this paper; In order to meet the basic physiological needs of accommodation, consumers generate external incentives for consumption. Second, the hotel experience value includes the internal motivation of hotel tenants and the corresponding emotional value. Third, in the process of the impact of experience value on customer satisfaction, which dimension of experience value is more critical to the impact of behavior results? Are there differences in different types of hotels? Therefore, this study takes the cognitive evaluation theory as the basis to explore the relationship between experience value and satisfaction and tries to analyze and verify the relationship between different dimensions of experience value and satisfaction.

Stimulus organism response (S–O–R) theory is developed from the stimulus response theory of behaviorism psychology. Stimulus response theory only analyzes external stimuli and action results. In order to study the internal perception and psychological state of stimulus recipients, scholars further put forward the stimulus organism response theory. S–O–R theory systematically explains how the external environment affects people's internal psychology and predicts people's subsequent behavior based on the response of this emotional attitude. It is a modern cognitive psychology theory about the relationship between external stimulation, individual attitude, evaluation, and subsequent behavior [14, 15]. Under the guidance of this theory, this paper analyzes the impact of experience value on satisfaction, regards the consumption process of customers in the hotel as an external stimulus, takes the resulting experience value as a bridge for communication stimulation and response, and takes customer satisfaction as the final result, and constructs the S–O–R theoretical model, as shown in Figure 6.

The article "Analyzing the Relationship between Hotel Brand Image, Service Quality, Experience Marketing, and Customer Satisfaction under the Environment of Social Network" was retracted in 2023. Reasons: unreliable results or conclusions; concerns about the data; concerns about the peer review; concerns about the citations.

### 3.3. Emotional Analysis of Experience Value

There are three mining methods of “feature viewpoint pair”: statistical method, semantic method, and domain ontology method. According to the research content of this paper, the “feature view pair” is extracted by statistical method, the Related words of different experience value dimensions are used as features, and the “feature view pair” is identified according to the proximity principle and certain view word matching rules; The weight of <f, o> matching is expressed by weight. When the weight reaches the threshold, it is considered that <f, o> matches and the viewpoint words are extracted correctly. After extracting the “feature viewpoint pair” of each sentence by statistical method, we need to use the emotion dictionary matching method to classify the emotion of different dimensions of experience value. The specific situation is shown in Table 1.

After identifying the “feature viewpoint pair” and giving the intensity value to the constructed emotion dictionary, respectively, the emotion of all 61206 effective online comments is analyzed. Based on the statistical method, this paper calculates the emotional scores of different dimensions of experience value in each comment. The calculation rules are shown in Table 2. Among them, EV represents the emotional value of different dimensions of experience value, *f* represents the intensity value of emotional words, *m* represents the number of adverbs, advisor represents the intensity value of adverbs, *n* represents the number of negative words, and *w* (Prij) represents the weight function of negative words. If the comment does not mention the characteristic words and emotional words of a certain dimension, it indicates that the customer's emotional attitude towards this dimension is neutral, that is, EV = 0 [16, 17].

According to Table 2, *i* is the comment number, *j* is the dimension of experience value, score 2 represents positive results, score 0 represents neutral, and score negative represents negative results, as shown in Table 3.

## 4. Result Analysis

According to the impact of brand community experience on user loyalty, the previous research object of the virtual brand community is mainly the electronic product community dominated by men, while the research object of a community dominated by women is relatively scarce, considering the importance of women in social networking and online shopping. Therefore, this study selected community users of make-up, clothing, tourism services, and snacks as the survey objects. A total of 200 questionnaires were randomly distributed, and 163 were recovered, including 132 valid questionnaires, with an effective questionnaire recovery rate of 80.9%. There are 24 items in the presurvey questionnaire and 132 valid questionnaires. The number of presurvey samples is 5.5 times that of the scale, which meets the requirements of the pretest samples of exploratory research [18, 19].

The article "Analyzing the Relationship between Hotel Brand Image, Service Quality, Experience Marketing, and Customer Satisfaction under the Environment of Social Network" was retracted in 2023. Reasons: unreliable results or conclusions; concerns about the data; concerns about the peer review; concerns about the citations.

### 4.1. Description and Analysis

Descriptive statistical analysis was conducted on the effective samples of the presurvey. In terms of gender (as shown in Figure 7 below), men accounted for 37% of the valid sample, and women accounted for 63% of the valid sample.

In terms of age (as shown in Figure 8 below), the number of people aged 21–30 ranks first among the effective samples, accounting for 43%; The number of people aged 31–40 accounted for the second in the effective sample, accounting for 32%; The number of people aged 41–50 accounted for the third in the effective sample, accounting for 16%.

In the presurvey valid samples, in terms of education level (as shown in Figure 9 below), the number of undergraduates ranks first in the valid samples, accounting for 36%; The number of junior college students is second in the effective sample, accounting for 30%; The number of graduate students is the third in the effective sample, accounting for 15%.

Among the presurvey valid samples, in terms of monthly income (as shown in Figure 10 below), the number of people with 5001–6000 yuan ranks first in the valid samples, accounting for 22%; 4001–5000 yuan, accounting for the second place in the effective sample, accounting for 20%; The number of effective samples is 6001–7000, accounting for 15%.

In the presurvey valid samples, in terms of work units (as shown in Figure 11), the number of other units ranks first in the valid samples, accounting for 32%; The number of private enterprises ranked second in the effective sample, accounting for 25%; The number of state-owned enterprises ranked third in the valid sample, accounting for 13%.

### 4.2. EF Analysis

Factor analysis is a very practical statistical technique in modern statistics. It includes two kinds of analysis: exploratory factor (EF) analysis and confirmatory factor (CF) analysis. This paper will conduct exploratory research on each variable from the following aspects, such as eigenvalue, cumulative variance contribution percentage, and so on. Factor analysis was conducted on 9 measurement items of virtual brand community experience. The eigenvalue results of the first-order factor analysis of virtual brand community experience are shown in Table 4.

The article "Analyzing the Relationship between Hotel Brand Image, Service Quality, Experience Marketing, and Customer Satisfaction under the Environment of Social Network" was retracted in 2023. Reasons: unreliable results or conclusions; concerns about the data; concerns about the peer review; concerns about the citations.

The EF analysis results of the presurvey effective sample data show that the reliability of each first-order factor is good, and the measurement items of each variable can fully explain themselves. This study will retain the original measurement items of these variables. Based on the analysis results of presurvey data, this study will conduct a formal survey and confirmatory factor analysis according to formal valid samples. According to the indicators shown in Figure 12, the formula is adopted:

(1) $$\begin{array}{c} P_{c}=\frac{{\left(\sum \lambda_{i}\right)}^{2}}{{\left(\sum \lambda_{i}\right)}^{2}+\left(\sum \varepsilon_{i}\right)}\left(1\right),\\ P_{v}=\frac{\sum \lambda_{i}^{2}}{\sum \lambda_{i}^{2}+\sum \varepsilon_{i}}\left(2\right), \end{array}$$

where *i* is the standardized load coefficient of the i-th observation variable, and *i* is the measurement error of the i-th observation variable. Among the three variables of the first-order model of brand community experience, the construction reliability *c* value of information experience (XE) is 0.8201 and the average variance extraction estimation v value is 0.6047, which is greater than the critical value, indicating that the internal consistency of the first-order measurement model of virtual brand community experience has passed the test.

## 5. Data Analysis and Suggestions

This chapter will build a regression model of the impact of experience value on satisfaction, use Eviews 10.0 to process the data of the model, and explore the impact of different dimensions of experience value on satisfaction. Firstly, starting with all hotel types, this paper analyzes the impact of different dimensions of customer experience value on satisfaction in the hotel industry; Then, it makes a regression analysis on the impact of different dimensions of customer experience value on the satisfaction of star hotels, economy hotels, and youth hostels; Finally, according to the research results, put forward more reasonable and effective suggestions to improve customer experience value and satisfaction [20].

### 5.1. Data Analysis

This section makes a quantitative analysis of the impact of different dimensions of experience value on satisfaction from the perspective of the whole and part by establishing a regression model. (1) The influence of the hotel's economic value, the hotel's emotional value, and the hotel's environmental value, (4) the degree of the hotel's economic value, the hotel's emotional value, and the hotel's social value, respectively. The degree of influence of functional value, economic value, situational value, emotional value, and social value of customer experience value on satisfaction.

The article "Analyzing the Relationship between Hotel Brand Image, Service Quality, Experience Marketing, and Customer Satisfaction under the Environment of Social Network" was retracted in 2023. Reasons: unreliable results or conclusions; concerns about the data; concerns about the peer review; concerns about the citations.

#### 5.1.1. Correlation Coefficient

The correlation coefficient of the variable is used to indicate the degree of correlation between the two variables, and the value is between -1 and 1. Taking the star rating as the dependent variable and the emotional scores of functional value, economic value, situational value, emotional value, and social value as the independent variables, this paper obtains the correlation coefficient table shown in Table 5. The correlation coefficient between variables is between 0.016 and 0.273, indicating that although there is a positive interaction between the five dimensions of experience value, the correlation coefficient is small, and the degree of this interaction is low.

According to the correlation coefficient, the variance inflation factor (VIF) between explanatory variables can be calculated. Vif is a measure of the degree of multicollinearity in a multiple regression model. The larger the Vif, the more serious the collinearity is. When <10, there is no multicollinearity between explanatory variables; When 10 ≤ Vif <100, there is strong multicollinearity; Vif ≥100, with severe multicollinearity. The specific calculation method is as follows: *VIF*=(1/1 − *R*_*i*_^2^)*R*_i_^2^ represents the correlation coefficient between the independent variable Xi and other independent variables during regression analysis. In this paper, it represents the correlation coefficient between the i-th dimension of experience value and other dimensions. The variance expansion factor between different dimensions of experience value is obtained according to the formula. Therefore, it is judged that there is no obvious multicollinearity between the experience values of different dimensions, and it is reasonable and effective to use the existing data for in-depth regression analysis.

#### 5.1.2. Regression Model

*(1) Econometric Model*. Emotional analysis obtains the emotional scores of consumers on different dimensions of experience value in each comment, indicating the emotional attitude of consumers. However, whether the specific dimensions of experience value have the same impact on consumer satisfaction and which aspects of experience consumers pay more attention to, there is a need to further establish a regression model for research. In this paper, the star rating of the hotel by customers is selected as the measurement index of customer satisfaction and as the explained variable. See the formula for details:

(2) $$\begin{array}{c} CSD=a_{1}Func+a_{2}Econ+a_{3}Sitn+a_{4}Emon+a_{5}Soc+u. \end{array}$$

In this measurement model, the explained variable CSD represents customer satisfaction, which is expressed by the star rating of customers on this consumption. The explanatory variable Func represents customers' perception of functional value, which is measured by the emotional score of functional value; Econ refers to customers' perception of economic value, which is measured by the emotional score of economic value; Sitn refers to customers' perception of situational value, which is measured by the emotional score of situational value; Emon refers to the customer's perception of emotional value, which is measured by the emotional score of emotional value; SOC refers to customers' perception of social value, which is measured by the emotional score of social value. I is the coefficient to be estimated of each dimension vector of experience value, and *u* is the random error term. Use Eviews 10.0 to process the data of the constructed regression model and obtain the model results [21].

*(2) Full Sample Regression*. Through the full sample regression of all comments in the hotel industry, it is found that the regression coefficients of explanatory variables have passed the significance test, which shows that all dimensions of experience value have a significant positive impact on customer satisfaction and show an obvious correlation. The regression equation under the whole sample is obtained according to model (1):

(3) $$\begin{array}{c} CSD=0.3147Func\left(22.8980\right)+0.6460Econ\left(31.2818\right)+0.7165Sitn\left(38.7749\right)+0.665Emon\left(39.9410\right)+0.4445Soc\left(17.9083\right)+u. \end{array}$$

The four thresholds are *γ*1 = −2., *γ*2 = −1.5730, *γ*3 = −0.6075, *γ*4 = 0.6608.

The article "Analyzing the Relationship between Hotel Brand Image, Service Quality, Experience Marketing, and Customer Satisfaction under the Environment of Social Network" was retracted in 2023. Reasons: unreliable results or conclusions; concerns about the data; concerns about the peer review; concerns about the citations.

According to the impact of different experience value dimensions on customer satisfaction, consumers pay more attention to subjective feelings. Only by providing a complex set of integrated products such as hotel facilities, atmosphere, and services at the same time can we meet the needs of tenants. The results show that when guests stay in the hotel, in addition to purchasing the right to use hotel rooms and other facilities, it is more important to enjoy the service. The connection and communication between people and the environment have a stronger impact on customer satisfaction.

### 5.2. Management Suggestions

The empirical results show that situational value has the most significant impact on customer satisfaction, which shows to a certain extent that allowing customers to enjoy a high standard of situational value experience and creating a unique hotel environment atmosphere is the key to enhancing the competitiveness of the hotel; Economic value is mainly reflected in consumers' overall perception of costs and benefits. People will always compare whether their pay and harvest are proportional or biased to one side, which requires hotel operators to improve consumers' perception of economic value from two aspects, which is not only the requirement for economic hotels and youth hostels but also applicable to star hotels. Try to reduce the cost of customers, mainly to reduce the cost of accommodation, and optimize the allocation by improving the operation efficiency of the enterprise and integrating resources; Functional value has a weak impact on customer satisfaction, which is the least significant dimension for the whole hotel industry, star hotels, and youth hostels. The hotel needs to build intelligent rooms to promote the realization of functional value; We should also carry out an online evaluation based on customer experience, pay attention to consumers' online comments, respond to customers' criticisms and opinions, and actively rectify them.

The article "Analyzing the Relationship between Hotel Brand Image, Service Quality, Experience Marketing, and Customer Satisfaction under the Environment of Social Network" was retracted in 2023. Reasons: unreliable results or conclusions; concerns about the data; concerns about the peer review; concerns about the citations.

## 6. Conclusion

Based on the online comments of the hotel industry, this paper studies the impact of customer experience value on satisfaction by using the methods of emotional analysis and econometric model and obtains the following conclusions: through combing and summarizing the relevant theories, it is found that the impact of experience value on satisfaction has reached a consensus; Most of the relevant studies focus on the service industry, but few studies explore the impact of different dimensions of experience value on satisfaction and then take targeted improvement measures. Using the method of manual marking to identify the characteristic words of different dimensions of experience value, build an emotion dictionary and give the intensity value. On the above basis, python programming is used to analyze the emotion of the comment text, and the emotion scores corresponding to different dimensions of experience value of each comment are obtained. Taking the star rating of the hotel as the measurement index of customer satisfaction as the explained variable and the emotional score of each dimension of experience value as the measurement index of customer experience value as the explanatory variable, an ordered logistic regression model is constructed. It is hoped that hotel operators can identify customer needs, allocate resources more effectively, and improve customer satisfaction from the perspective of improving customer experience according to their own hotel type and market positioning.

Under the guidance of relevant theories, this paper selects 61206 effective online comments on a platform as the research object to analyze the impact of customer experience value on satisfaction in the hotel industry. There are some deficiencies in the research process, which need to be further improved in the following aspects:

1. Diversified sample selection. This paper selects the online comments of different types of hotels in Qingdao as the research object, and consumers in different cities may have different concerns. In future research, we can select the online comments of multiple cities for comparative analysis to get more comprehensive and perfect results.
2. Add control variables. In this paper, the hotel industry is selected as the research object, which is divided into three different hotel types for heterogeneity analysis. In future research, we can choose the variables that show the characteristics of customer behavior, such as travel purpose, as the control variables, analyze the impact of each dimension of experience value on different types of travel people, and more clearly understand the needs of different types of customers, and guide the behavior of hotel operators.

The article "Analyzing the Relationship between Hotel Brand Image, Service Quality, Experience Marketing, and Customer Satisfaction under the Environment of Social Network" was retracted in 2023. Reasons: unreliable results or conclusions; concerns about the data; concerns about the peer review; concerns about the citations.

## Figures and Tables

**Figure 1:** Four cores of community operation.

**Figure 2:** Customer experience measurement model of brand community.

**Figure 3:** Customer experience-brand loyalty model.

**Figure 4:** Antecedent model of brand loyalty.

**Figure 5:** Customer satisfaction model.

**Figure 6:** S–O–R model diagram.

**Figure 7:** Sex ratio of exploratory research samples.

**Figure 8:** Age distribution of exploratory research samples.

**Figure 9:** Education level of the exploratory research sample.

**Figure 10:** Monthly income of exploratory research sample.

**Figure 11:** Work units of exploratory research samples.

**Figure 12:** First-order measurement model of brand community experience and its output results.

**Table 1:** Dictionary and intensity of experience value and emotion in the hotel industry.

Dictionary	Strength value	Examples
Positive basic emotion dictionary	1.0	Good, great, excellent, OK, perfect
Dictionary of negative basic emotions	−1.0	Bad, rotten, regret, complain
Positive hotel experience value	1.0	Convenient, prosperous, tidy, cost-effective, and value for money
Special emotion dictionary	−1.0	Comfortable, diligent, and considerate
Negative word	−1.0	No, never, cannot, very little
	2.0	Most, extremely, completely, absolutely, super
	1.5	Especially, very, real, more
Adverb of degree	1.0	Comparison, more
	0.5	A little, some, pretty

**Table 2:** Rules for calculating emotional scores.

Text type	Formula	Examples
Not mentioned	EV = 0	
Characteristic words		
Feature words + emotional words	EV = *f* (x)	Cost-effective
Feature word + adverb + emotion word	*EV*=*fx*∏_*i*=1_^*m*^*A* *dv*_*i*_	Poor sound insulation
Characteristic words + negative words + emotional words	*EV*=*fx*∏_*j*=1_^*m*^*w*Pr*i*_*j*_	Service attitude was not friendly
Characteristic word + negative word + adverb + emotional word	EV = *f* (x)	The location is not remote
	∏_*i*=1_^*m*^*A* *dv*_*i*_∏_*i*=1_^*m*^*w*Pr*i*_*j*_	

The article "Analyzing the Relationship between Hotel Brand Image, Service Quality, Experience Marketing, and Customer Satisfaction under the Environment of Social Network" was retracted in 2023. Reasons: unreliable results or conclusions; concerns about the data; concerns about the peer review; concerns about the citations.

**Table 3:** Emotional scores of experience value.

Comment	Experience value emotion score				
	EVij (*j* = 1)	EVij (*j* = 2)	EVij (*j* = 3)	EVij (*j* = 4)	EVij (*j* = 5)
*i* = 1	2	0	0	−1	0
*i* = 2	1.5	1	−1.5	1	0
*i* = 3	1	0	1.5	0	−1
...	...	...	...	...	...
*i* = 61204	1.5	1.5	1	1	1

**Table 4:** Eigenvalues of first-order factor analysis of brand community experience.

Factor	1	2	3
Characteristic quantity	4.484	1.823	1.079

**Table 5:** Correlation coefficient.

Variable	Star rating	Func	Econ	Sitn	Emon	Soc
Star rating	1	0.187	0.223	0.234	0.268	0.123
Func		1	0.171	0.111	0.263	0.015
Econ			1	0.052	0.172	0.039
Sitn				1	0.071	0.101
Emon					1	0.071
Soc						1

## Data Availability

The labeled dataset used to support the findings of this study is available from the author upon request.
